The article "Efficacy Evaluation of the VFQ-25 Scale in Patients with Different Degrees of Vitreous Opacity After Nd : YAG Laser Ablation" was retracted in 2023. Reasons: signs of a paper mill; suspected computer-generated content; unreliable results or conclusions; concerns about the data.

# Efficacy Evaluation of the VFQ-25 Scale in Patients with Different Degrees of Vitreous Opacity After Nd : YAG Laser Ablation

**DOI:** 10.1155/2022/5075447

**Published:** 2022-09-28

**Authors:** Siwei Zhang, Kang Yang, Bin Wang

**Affiliations:** ^1^Department of Ophthalmology, Hefei Bright Eye Hospital, Hefei 230001, Anhui, China; ^2^Department of Ophthalmology, Fuyang Women and Children's Hospital, Fuyang 236000, Anhui, China

## Abstract

**Objective:**

To evaluate the effect of the VFQ-25 scale on the efficacy of Nd : YAG laser ablation in patients with different severity of vitreous opacities.

**Methods:**

From January 2020 to March 2021, data of patients who presented to our department and were diagnosed with vitreous opacity were collected, and the severity of vitreous opacity was divided into four grades: I, II, III, and IV. Preoperative visual acuity, intraocular pressure, dilated fundus, B ultrasound, and other examinations were performed, and the patients were scored using the VFQ-25 scale. All patients underwent Nd : YAG laser ablation and were followed for 6 months. The VFQ-25 scale was again used postoperatively to score the patient's efficacy. The general information and clinical characteristics of the patients we collected. The Spearman's test was used to evaluate the correlation between VFQ-25 score and Nd : YAG laser efficacy in patients.

**Results:**

A total of 80 patients (95 eyes) were included in this study. Vitreous opacities were grade I in 56 eyes (58.9%), grade II in 22 eyes (23.2%), grade III in 10 eyes (10.5%), and grade IV in 7 eyes (7.4%). Compared with preoperative scores, patients with vitreous opacity had significantly higher postoperative scores in terms of overall health (36.54 ± 17.06 vs 33.52 ± 16.74), overall visual acuity (60.39 ± 14.24 vs 57.56 ± 13.13), color vision (88.94 ± 12.56 vs 86.38 ± 12.37), and peripheral visual acuity (74.06 ± 18.38 vs 72.20 ± 18.79) items (all *P* < 0.001). The overall response rates of vitreous opacities I, II, III, and IV were 100%, 90.9%, 80.0%, and 71.4%, respectively. There was a significant correlation between the postoperative VFQ-25 total score, and the therapeutic effect of laser ablation for grade I vitreous opacities, with a correlation coefficient *r* of 0.417 (*P*=0.001). The correlation coefficient *r* between the total score of postoperative VFQ-25 and the treatment effect of grade II vitreous opacity was 0.622 (*P*=0.002). However, the correlation between the postoperative efficacy of grade III and IV patients and the VFQ-25 score was not significant.

**Conclusion:**

In patients with different degrees of vitreous opacity undergoing Nd : YAG laser vitreous ablation, the overall health, overall visual acuity, color vision, and peripheral visual acuity were improved after surgery, and the VFQ-25 score was significantly correlated with the postoperative efficacy, which is worthy of clinical use.

## 1. Introduction

The vitreous body is an extracellular matrix consisting of 98% water and macromolecules, the most important of which are hyaluronic acid and collagen in clear gel [1]. The vitreous structure changes caused by aging, inflammation, vitreoretinal dystrophy, diabetic vitreous disease, or myopia. The homogeneity of the vitreous decreases, and even formed elements will be precipitated, forming floating opacities such as dust and cloud floccules, that is, vitreous opacities [2]. Emerging evidence suggests that perception of vitreous opacities and associated visual disturbances are more prevalent than once thought [3]. Nd : YAG laser ablation is a new technology that has rapidly developed since the 1980s. It first achieved varying degrees of success in the treatment of posterior ocular diseases, while in recent years, the use of Nd : YAG laser ablation for vitreous opacities has attracted much attention [4]. In general, Nd : YAG laser ablation is safe, but it still does not seem to benefit all patients [5]. A scale, or marker, is needed to evaluate the efficacy of Nd : YAG laser ablation for vitreous opacities. The VFQ-25 scale is a practical tool for assessing visual function and vision-related quality of life and not only reflects disease status but also includes factors that affect quality of life, such as mental status, and social functioning [6]. Currently, there are still a few studies using the VFQ-25 scale to evaluate the efficacy of Nd : YAG laser ablation in patients with different severity of vitreous opacities. The aim of this study was to assess the correlation between the VFQ-25 scale and treatment outcome by analyzing vitreous opacities treated with a 1064 nm neodymium : yttrium-aluminum-garnet laser (Nd∶ YAG laser).

## 2. Objects and Methods

### 2.1. Objective

From January 2020 to March 2021, the data of 95 eyes of 80 patients (28 males and 52 females, mean age 58 ± 12 years) who presented to our department and were diagnosed with vitreous opacity were collected.

Inclusion criteria is as follows: (1) vitreous opacity was confirmed by B ultrasound and slit lamp examination; (2) there were dust and cloud flocculent floaters in front of the eyes and affected life; and (3) the general health status was stable, and the symptoms were stable within half a year.

Exclusion criteria is as follows: (1) previous history of ocular surgery; (2) ocular diseases with uveitis, fundus lesions, and other ocular diseases affecting treatment or causing complications; (3) risk of retinal detachment; (4) unable to cooperate, or failed to adhere to treatment and follow-up; and (5) combined liver and kidney dysfunction, tumors or bleeding, and coagulation diseases. All patients were informed and signed a consent form. The study protocol was approved by the Ethics Committee of Hefei Bright Eye Hospital.

### 2.2. Severity Grading for Vitreous Opacities

Grade I refers to discomfort during vision, and monomeric opacities can be seen in the fundus; grade II refers to discomfort during vision, and several clear monomeric opacities can be seen in the fundus; grade III refers to obvious symptoms, an annular floating sensation during vision, and obvious annular opacities can be seen in the fundus; and grade IV refers to obvious symptoms, nebulous discomfort during vision, and a large number of opacities of different shapes can be seen in the fundus.

## 3. Method

### 3.1. Treatment Methods

All patients underwent visual acuity, intraocular pressure, dilated fundus, and B ultrasound. The Lumenis SmartV Selecta Duet Laser System was selected for laser treatment with parameters set to a starting energy of 2.0–8.0 mJ, single point emission, and energy parameters were progressively adjusted to vaporize the opacities. During the treatment, the number of pulses emitted per treatment is controlled within 500, and the time is controlled within 30 minutes according to the previous order after up and down. If there are still many opacities, elective retreatment is carried out.

### 3.2. Follow-up and Efficacy Determination

All patients were followed up until 6 months after laser treatment. Visual acuity, intraocular pressure, dilated fundus, and B ultrasound were re-examined to analyze the improvement of clinical symptoms. Criteria for curative effect determination is as follows: (1) markedly effective: the symptoms disappeared, and no complications were observed; (2) effective: the symptoms were improved, and no complications were observed; (3) ineffective: the symptoms were not improved, with or without complications. Overall response rate = (markedly effective + effective)/total number of eyes × 100%. The complications include lens injury, postoperative high intraocular pressure, glaucoma, retinal hemorrhage, and an increased number of floating objects.

### 3.3. Statistical Analysis

Continuous variables were presented as mean ± standard deviation, and a paired *t*-test was used to compare differences in the VFQ-25 scores before and after laser treatment in patients with vitreous opacities. Categorical variables were presented as frequencies (percentages) and differences in overall response rates among patients with different severity of vitreous opacities were assessed by the chi-square test. The Spearman's test was used to evaluate the correlation between VFQ-25 score and Nd : YAG laser efficacy in patients. Two-sided *P* < 0.05 was considered statistically significant. Data were analyzed using SPSS statistics 21.0 (IBM SPSS, Armonk, NY).

## 4. Results

### 4.1. Baseline Characteristics

As shown in Table 1, a total of 80 patients and 95 eyes were included in this study. The average age of patients was 58 ± 12 years, 65.0% (52/80) were female, and 18.8% (15/80) had a history of diabetes. Among the causes of vitreous opacity, posterior vitreous detachment accounted for 72.6% (69/95), vitreous liquefaction degeneration 16.8% (16/95), and high myopia 10.5% (10/95). In terms of severity grading, 56 eyes (58.9%) had grade I vitreous opacity, 22 eyes (23.2%) had grade II vitreous opacity, 10 eyes (10.5%) had grade III vitreous opacity, and 7 eyes (7.4%) had grade IV vitreous opacity.

### 4.2. VFQ-25 Score before and after Surgery

As shown in Table 2, compared with preoperative scores, patients with vitreous opacity had significantly higher postoperative scores for the items of general health (36.54 ± 17.06 vs 33.52 ± 16.74), overall visual acuity (60.39 ± 14.24 vs 57.56 ± 13.13), color vision (88.94 ± 12.56 vs 86.38 ± 12.37), and peripheral visual acuity (74.06 ± 18.38 vs 72.20 ± 18.79) (*P* < 0.001). However, the preoperative and postoperative scores of near vision activity, distance vision activity, social function, mental health, social activity role disorder, eye pain, social dependence, and driving were similar, and the differences were not statistically significant (*P* > 0.05).

### 4.3. Laser Treatment Effectiveness

As shown in Table 3, the significant rate of grade I vitreous opacity was 76.8%, the total effective rate was 100%, the significant rate of grade II vitreous opacity was 68.2%, the total effective rate was 90.9%, the significant rate of grade III vitreous opacity was 30.0%, the total effective rate was 80.0%, the significant rate of grade IV vitreous opacity was 14.3%, and the total effective rate was 71.4%. For vitreous patients of different grades, the overall response rate after laser treatment was different, and the difference had statistical significance (*χ*^2^ = 22.576, *P*=0.001).

Correlation of VFQ-25 with Treatment Effect.

As shown in Table 4, the postoperative total VFQ-25 score was significantly correlated with the therapeutic effect of laser ablation for grade I vitreous opacities, with a correlation coefficient *r* of 0.417 (*P*=0.001). The correlation coefficient *r* between the total score of postoperative VFQ-25 and the treatment effect of grade II vitreous opacity was 0.622 (*P*=0.002). The correlation coefficient *r* between the postoperative VFQ-25 score and the treatment effect of grade III vitreous opacity was 0.583 (*P*=0.077). The correlation coefficient *r* between the postoperative VFQ-25 score and the treatment effect of grade IV vitreous opacity was 0.673 (*P*=0.097).

## 5. Discussion

In patients with vitreous opacities, Nd: YAG laser ablation was found to significantly improve overall health, overall visual acuity, color vision, and peripheral visual acuity item scores. Different severity of vitreous opacity may lead to different therapeutic effects. Notably, the postoperative VFQ-25 score was significantly correlated with the treatment effect of laser ablation.

Vitreous opacity is most commonly caused by posterior vitreous detachment, and a small proportion can also be caused by vitreous liquefaction deformation and high myopia, and vitreous opacity can lead to blurred vision and decreased visual acuity [7]. Even if these symptoms are considered nonpathological, they may affect quality of life and mood for many patients and myopic patients with posterior vitreous detachment are more sensitive to these symptoms. Vitreous opacities that do not affect vision and daily life generally do not require treatment or administration of medication. For symptomatic patients with vitreous opacities, Nd : YAG laser vitreolysis may be a treatment option [8]. This treatment technique is noninvasive and allows precise localization of floaters within the vitreous cavity through a special optical lens followed by vaporization and ionization vaporization to form small molecular valorization gases such as CO, H2, CH4, and other gases to facilitate absorption, thereby treating vitreous opacities and improving patient symptoms [9].

Studies have shown that among patients with vitreous opacities undergoing Nd : YAG laser vitrectomy, 75% reported significant improvement and 25% reported moderate improvement [10]. This is in general agreement with our findings, where the overall response rate was 100% in patients with vitreous opacities of grade I and 71.4%–90.9% in patients with grades II–IV. Therefore, Nd : YAG laser vitrectomy is well-tolerated and effective treatment for vitreous opacities. In using this technique, the following points of attention are also required. First, the laser is confined to the middle and posterior vitreous. Anterior vitreous opacification has little impact on visual quality and visual acuity, but retinal and posterior lens capsule damage needs to be avoided, with a safe distance of 3–4 mm anterior to the retina and 2–3 mm posterior to the lens, and the operation is prohibited directly in front of the fovea, with a maximum energy of <8.0 Mj [11]. Second, the operating physician should pay attention to the movement of vitreous opacity to avoid laser action on the retina [5]. Third, specially designed convex contact lenses should also be used to lower the energy threshold for plasma formation and improve the safety of intravitreal YAG lasers [12].

The VFQ-25 score was developed with support from the National Eye Institute to create a survey measuring self-reported sight-targeted health status and further incorporate the impact of quality of life, such as emotional well-being and social functioning [13]. The VFQ25 score, which consists of 25 questions, has been widely used for glaucoma, cataracts, diabetic retinopathy, and low-vision diseases due to various causes [13]. In this study, the VFQ-25 score was used for the first time to evaluate the therapeutic effect of Nd : YAG laser vitrectomy in patients with vitreous opacity, and the results suggested that in patients with vitreous opacity, Nd: YAG laser ablation could significantly improve the scores of overall health, overall visual acuity, color vision, and peripheral visual acuity items.

Symptoms such as blurred vision and impaired vision are the main factors afflicting patients with vitreous opacity, but they also have further life and work impact. Previous studies have shown that the VFQ-25 score is a good scale for evaluating the severity of symptoms in patients with vitreous opacities and has reliable reliability and validity [14]. The VFQ-25 scale shows high internal consistency (Cronbach *α* range 0.739–0.932) and high test-retest reliability (intraclass correlation coefficient 0.876–0.975) [15]. This study also found that the VFQ-25 score was significantly associated with the treatment effect of laser ablation and could be used to evaluate the efficacy of laser ablation.

However, this study also has the following limitations: the study had a small sample size, no treatment control group was set and only the treatment effect at 6 months after surgery was observed in this study. In addition, we observed a significant correlation between the VFQ-25 score and postoperative efficacy in patients with grade I and II vitreous opacity. However, we did not observe a significant correlation in patients with grades III and IV, which may be related to our small sample size. Future large, prospective randomized controlled clinical trials are needed to evaluate the role of the VFQ-25 score in patients undergoing laser ablation for vitreous opacities.

In summary, in patients with different degrees of vitreous opacity undergoing Nd : YAG laser vitreous ablation, the VFQ-25 score was significantly correlated with the postoperative efficacy, which is worthy of clinical use.

## Figures and Tables

**Table 1:** Clinical characteristics of patients with vitreous opacity.

	Patients with vitreous opacity
Number, *n*	80
Number of eyes, *n*	95
Age, years	58 ± 12
Proportion of females, *n* (%)	52 (65.0)
History of diabetes, *n* (%)	15 (18.8)
Causes of vitreous opacity	
Posterior vitreous detachment	69 (72.6)
Vitreous liquefaction degeneration	16 (16.8)
High myopia	10 (10.5)
Severity grade	
Grade I	56 (58.9)
Grade II	22 (23.2)
Grade III	10 (10.5)
Grade IV	7 (7.4)

**Table 2:** VFQ-25 scores of patients with vitreous opacity before and after operation.

Item	Preoperative score	Post OPERATIVE SCORE	*P* Value
General health	33.52 ± 16.74	36.54 ± 17.06	<0.001
Overall visual acuity	57.56 ± 13.13	60.39 ± 14.24	<0.001
Near vision activity	72.07 ± 11.86	70.71 ± 12.18	0.147
Distance vision activity	55.45 ± 15.34	57.01 ± 15.56	0.219
Social functioning	72.87 ± 15.43	72.29 ± 13.73	0.742
Mental health	48.94 ± 15.59	47.61 ± 13.44	0.417
Role disorder in social activities	47.59 ± 14.93	45.68 ± 14.99	0.249
Color vision	86.38 ± 12.37	88.94 ± 12.56	<0.001
Peripheral vision	72.20 ± 18.79	74.06 ± 18.38	<0.001
Eye pain	78.61 ± 11.98	77.58 ± 9.85	0.418
Social dependence	71.25 ± 14.50	69.58 ± 14.87	0.082
Driving	70.05 ± 15.15	68.71 ± 14.83	0.077

**Table 3:** The laser treatment effect in patients with different severity of vitreous opacity.

	Number of eyes	Markedly effective	Effective	Invalid	Overall response rate,%
Grade I, *n* (%)	56	43 (76.8)	13 (23.2)	0 (0)	100
Grade II, *n* (%)	22	15 (68.2)	5 (22.7)	2 (9.1)	90.9
Grade III, *n* (%)	10	3 (30.0)	5 (50.0)	2 (20.0)	80.0
Grade IV, *n* (%)	7	1 (14.3)	4 (57.1)	2 (28.6)	71.4
Χ^2^	22.576				
*P* Value	0.001				

**Table 4:** Correlation of the postoperative VFQ-25 total score with therapeutic effect of laser ablation.

	Correlation coefficient r	*P* Value
Grade I	0.417	0.001
Grade II	0.622	0.002
Grade III	0.583	0.077
Grade IV	0.673	0.097

## Data Availability

The analyzed data sets generated during the study are available from the corresponding author on reasonable request.
